# Speckle Noise Algorithm-Based Ultrasound Imaging in Evaluating the Therapeutic Effect of Blood Purification on Children with Kidney Failure and Analysis of Its Correlation with Serum Inflammatory Factor Levels

**DOI:** 10.1155/2022/3384102

**Published:** 2022-01-29

**Authors:** Xueqin Li, Hui Guo, Soinam Songjin, Ning Mo, Xiuying Chen

**Affiliations:** ^1^Department of Pediatrics Nephrology Nursing, West China Second University Hospital, Sichuan University/West China School of Nursing, Sichuan University, Chengdu 610041, Sichuan, China; ^2^Key Laboratory of Birth Defects and Related Diseases of Women and Children (Sichuan University), Ministry of Education, Chengdu 850002, Sichuan, China; ^3^Department of Pediatric Nephrology, The Second People's Hospital of Tibet Autonomous Region, Lhasa, Tibet Autonomous Region 610041, China; ^4^Department of Pediatric Nephrology, Chengdu Western Angel Child Maternity Hospital, Chengdu 610041, Sichuan, China

## Abstract

The study focused on the therapeutic effect of clinical treatment on urinary calculi with kidney failure and its relationship with the serum inflammatory factor levels. 90 children with melamine urinary calculi were selected as research subjects. Of them, 52 cases were in group 1 (nonrenal failure), and 38 cases were in group 2 (combined with renal failure). In addition, 35 hospitalized children with no history of melamine-contaminated milk feeding during the same period were used as healthy controls. They all underwent ultrasound imaging examination based on the speckle noise algorithm, and the prognosis was analyzed. It was found that the peak signal-to-noise ratio (PSNR), structural similarity (SSIM), and local edge preservation index (EPI) of the algorithm in this study were significantly greater than other algorithms (*P* < 0.05). The admission age of the children in group 1 was significantly younger than that of group 2, the bilateral stone rate was significantly higher than that in group 2, and the difference was statistically significant (*P* < 0.05). Of the 52 children in group 1, the stone disappeared in 25 cases after treatment, the stone was reduced in 20 cases, and the stone remained unchanged in 7 cases. The total effective rate of treatment was 88.46%. Of the 38 cases in group 2, the stone disappeared in 22 cases after treatment, the stone was reduced in 12 cases, and the stone remained unchanged in 4 cases. The total effective rate of treatment was 89.47%. No difference was noted in blood urea nitrogen (BUN), blood creatinine (Cr), TNF-*α*, and C-reactive protein (CRP) levels in group 1, group 2, and the healthy control group (*P* > 0.05). Hence, the denoising algorithm in this study has better denoising effects on ultrasound images than traditional algorithms, with higher definition and less noise and artifacts. The clinical treatment of children with urinary calculi and renal failure is highly effective, the renal function and serum inflammatory factor levels return to the normal range, and the inflammatory response is weakened.

## 1. Introduction

Kidney failure is a decline in kidney function that occurs when the kidneys are unable to maintain metabolism and water and electrolyte balance. Renal failure is divided into acute renal failure and chronic renal failure [1, 2]. Acute renal failure arises from the rapid decline of glomerular filtration rate, accumulation of nitrogenous waste in the body, water and sodium retention, and electrolyte imbalance, and patients will have symptoms such as reduced urine output or even anuria, general edema, and heart failure [3]. Acute renal failure is also known as acute kidney injury, and its causes include prerenal, renal parenchymal, and postrenal factors [4, 5]. Acute kidney injury caused by prerenal and postrenal factors is reversible but timely diagnosis and active treatment contribute to a good prognosis and in most cases can restore the kidney function to normal [6–8]. In clinical practice, chronic renal failure is common in nephrology, mainly arising from kidney damage and serious destruction of the nephron, which then lead to endocrine disorders, nitrogen metabolite storage disorders, and water electrolyte and acid-base balance disorders. In the case of chronic renal failure, the body's immunity and resistance will decrease significantly, and the internal environment disorders caused by renal excretion and metabolic dysfunction will further make the body's response to infection abnormal. Worse still, the clinical application of antibiotics is subject to various limitations [9]. Clinical treatment of acute renal failure and chronic renal failure generally uses hemodialysis. Hemodialysis is a renal replacement treatment for patients with acute and chronic kidney failure. It can drain blood from the body to the outside of the body and pass it through a dialyzer composed of countless hollow fibers. The electrolyte solution (dialysis solution) with a similar concentration of the blood exchanges substances with the blood to remove metabolic waste, maintain electrolyte and acid-base balance, and at the same time remove the excessive water [10]. In the study, hemodialysis was performed on children with urinary stones and renal failure.

With the continuous advancement of science and technology, medical ultrasound imaging technology has made great progress in both imaging quality and imaging speed [11]. Ultrasound has become one of the commonly used examination methods for kidney diseases due to its advantages of noninvasiveness, convenience, low cost, and reproducibility, and whether there are congenital malformations, cystic lesions, and stones can be determined by observing the shape of the kidney. In the meanwhile, it can also be used for the auxiliary examination of acute renal failure [12, 13]. However, due to the limitations of ultrasound imaging mechanisms, ultrasound images have inherent disadvantages. A large amount of speckle noise often appears in the original ultrasound image, reducing the readability, and it is impossible to observe the tiny structural edges and lesion areas, which increases the risk of misdiagnosis [14–16]. The removal of speckle noise in ultrasound images has always been a topic of great concern in the medical field. Traditional ultrasound image denoising techniques are mainly image filtering techniques in the spatial domain, such as classic median filtering, mean filtering, and Wiener filtering. However, these methods face an obvious contradiction between noise filtering and edge preservation, so they have certain limitations. Speckle noise algorithm solves the initial value of the partial differential diffusion equation of the original image and takes different diffusion coefficients and the numbers of iterations to generate the corresponding scale image and further produce the final filter image by image transformation. This kind of algorithm is not influenced by the filtering window and the shape. When applied to process ultrasonic images, it can effectively suppress noise while preserving image details and even enhance contrast and improve image quality, which can overcome the difficulties existing in traditional algorithms.

The study aimed to analyze the effect of clinical treatment of urolithiasis complicated with renal failure and the changes of serum inflammatory factors, expected to provide a reference for the clinical treatment of children with renal failure. Ninety children with melamine urinary calculi who were admitted to the hospital were selected as the research subjects. According to the presence or absence of renal failure, 52 cases were in group 1 (nonrenal failure), and 38 cases were in group 2 (combined with renal failure). They all underwent ultrasound imaging examination based on the speckle noise algorithm. The effect of clinical treatment was evaluated, factoring into the effective rate, prognosis, renal function, and changes in inflammatory factor levels. Additionally, the relationship between urinary calculi combined with kidney failure and serum inflammatory factor levels was analyzed.

## 2. Materials and Methods

### 2.1. Research Subjects

Ninety children with melamine urinary calculi who were admitted to the hospital from May 3, 2019, to January 15, 2021, were selected as the research subjects, including 53 males and 37 females. According to the presence or absence of renal failure, 52 cases were in group 1 (nonrenal failure), and 38 cases were in group 2 (combined with renal failure). In addition, 35 hospitalized children who had no history of drinking melamine-contaminated milk and were free of urinary tract diseases during the same period were selected as the healthy control group, including 23 males and 12 females. This study has been approved by the Medical Ethics Committee of the hospital, and the subjects and their family members fully understood the situation of the study and had signed an informed consent form.

Inclusion criteria were as follows: (I) children with complete clinical data; (II) children who had signed an informed consent form; (III) children under 3 years of age; (IV) imaging examination that confirmed the presence of urinary calculi; and (IV) hematuria examination showing normal red blood cell morphology. Exclusion criteria were as follows: (I) hematuria of glomerular origin; (II) children with urinary tract malformations; (III) children who withdrew from the experiment midway; and (IV) children with metabolic diseases.

### 2.2. Ultrasound Examination

Color Doppler ultrasound system was used to perform urinary tract ultrasound examination on the child with a probe frequency of 3.5 MHz. Before the examination, the child was allowed to drink a proper amount of water to fill the bladder. During the examination, the child was in a lateral position. The probe was placed in the double kidney area to scan the kidneys. Then, it walked along the renal hilum, renal pelvis, and ureter to check the junction of the renal pelvis and ureter and the upper part of the ureter. Next, in the supine position, the outer edge of the rectus abdominis was compressed. After the walking direction of the abdominal aorta was identified, the intestine was opened, and the probe walked along the ureter to scan the abdominal segment, pelvic segment, second stricture, and terminal segment of the ureter. Next, the bladder above the symphysis pubis was scanned, and the angle was adjusted to display the opening of the bilateral ureters in the bladder wall. Subsequently, the presence or absence of urinary calculi and the presence or absence of dilation of the collecting system of the kidneys and the ureter were observed. If there were urinary tract stones, the size, number, location, shape, and internal echo of the urinary tract were recorded, and it was checked whether there were urinary tract malformations.

### 2.3. Ultrasound Denoising Algorithm Based on Shearlet Transform and KDA Model

Shearlet transform (ST) [17] is a new type of multiscale geometric analysis tool. Compared with contourlet transform, it has lower time complexity and unlimited number of directions. However, ST does not have translation invariance, and the pseudo-Gibbs phenomenon will occur during image reconstruction. Therefore, in this study, the nonsubsampled shearlet transform (NSST) is introduced to optimize it.

First, the two-dimensional compound expansion affine system can be expressed as follows:

(1) $$\begin{array}{c} {ƛ}_{PQ}\left(\omega \right)=\left\{\omega_{i,j,n}\left(x\right){\left|\det P\right|}^{1/2}\omega \left(Q^{k}P^{i}x-n\right):i,k\in W,n\in W^{2}\right\}, \end{array}$$

where *P* and *Q* represent a 2 × 2 invertible matrix, |det *P*|=1, and both *n* and *k* are constants. If *ƛ*_*PQ*_(*ω*), there is

(2) $$\begin{array}{c} {\sum_{i,k,n}\left|\left(h,\omega_{i,k,n}\right)\right|}^{2}={\left\|h\right\|}^{2}. \end{array}$$

Then, the elements of the system are called composite wavelets. *P*^*i*^ is related to scale changes and *Q*^*k*^ is associated with geometric transformations with constant area. Let $P=\begin{array}{ccc} P_{0} & or & P_{1} \end{array}$, $Q=\begin{array}{ccc} Q_{0} & or & Q_{1} \end{array}$, $P_{0}=\langle \begin{array}{cc} 5 & 0\\ 0 & 3 \end{array}\rangle$, $P_{1}=\langle \begin{array}{cc} 3 & 0\\ 0 & 5 \end{array}\rangle$, $Q_{0}=\langle \begin{array}{cc} 2 & 2\\ 0 & 2 \end{array}\rangle$, and $Q_{1}=\langle \begin{array}{cc} 2 & 0\\ 2 & 2 \end{array}\rangle$; then, the set in (1) is a shear wave, $P=\begin{array}{ccc} P_{0} & \text{or} & P_{1} \end{array}$ is an anisotropic stretching matrix, and $Q=\begin{array}{ccc} Q_{0} & \text{or} & Q_{1} \end{array}$ is a shear matrix. Then, the shear wave transform function is as follows:

(3) $$\begin{array}{c} \omega_{i,k,n}^{\left(0\right)}\left(x\right)=2^{3i/2}\omega^{\left(0\right)}\left(Q_{0}^{k}P_{0}^{i}x-n\right),\\ \omega_{i,k,n}^{\left(1\right)}\left(x\right)=2^{3i/2}\omega^{\left(1\right)}\left(Q_{0}^{k}P_{0}^{i}x-n\right), \end{array}$$

where *i* ≥ 0, −2^*i*^ ≤ *k* ≤ 2^*i*^, *ω*^(0)^(*β*)=*ω*^(0)^(*β*_1_.*β*_2_)=*ω*_1_(*β*_1_)*ω*_2_(*β*_2_/*β*_1_), and *ω*^(1)^(*β*)=*ω*^(1)^(*β*_1_.*β*_2_)=*ω*_1_(*χ*_2_)*ω*_2_(*β*_2_/*β*_1_). For any (*β*_1_.*β*_2_) ∈ *C*_0_, *C*_0_={(*β*_1_.*β*_2_) ∈ *ℜ*^2^*|*|*β*_1_| ≥ 1/*Q*, |*β*_2_/*β*_1_| ≤ 1}, *C*_1_={(*β*_1_.*β*_2_) ∈ *ℜ*^2^*|*|*β*_1_| ≥ 1/*Q*, |*β*_2_/*β*_1_| ≤ 1} constitutes the supporting domain of *ω*_*i*,*k*,*n*_^(0)^(*x*) and *ω*_*i*,*k*,*n*_^(1)^(*x*).  Figure 1 shows the support frequency domain of the shear wave in the *ℜ*^2^ plane. The yellow line represents *C*_1_, and the green line represents *C*_0_.

Thus, for any image *hi* ≥ 0, −2^*i*^ ≤ *k* ≤ 2^*i*^, the ST can be expressed as follows:

(4) $$\begin{array}{c} {\text{Shearlet}}_{\omega }h_{{}_{\left(i,k,n\right)}}=\left(h,\omega_{i,k,n}^{\left(c\right)}\right). \end{array}$$

The NSST transform discretization constructs the algorithm together with the Laplacian pyramid and the directional filter [18]. First, the image is decomposed by the Laplacian pyramid to obtain a high-frequency subband and a low-frequency subband. The subband represents the edge detail information in the image, and the low-frequency subband represents the overview of the original image. Then, the high-frequency subband is divided by directions with a directional filter to obtain the directional detail information in the image. Next, the low-frequency subband is further decomposed, and the above steps are repeated (Figure 2).

The threshold function is weighted by scale to prevent the decrease of noise pollution level with the reduction of resolution [19], and the scale function controls the size of the threshold under the resolution to effectively filter out the noise under each resolution. Therefore, the scaling function is defined as follows:

(5) $$\begin{array}{c} W\left(r\right)=\sqrt{\alpha \;\log\left(\frac{r+1}{r}\right)}, \end{array}$$

where *r* represents the scale where the NSST transform coefficients are located, *r* = 1 represents high resolution, and *α* represents the attenuation degree parameter. Then, the hard threshold method is introduced for improvement, expressed as follows:

(6) $$\begin{array}{c} S_{i,j}=\theta W\left(r\right)\phi_{i},\phi_{j}, \end{array}$$

where *θ* is the constant that controls the global threshold, *W*(*r*) represents the scale weighting function, *ϕ* represents the standard deviation of the noise image, and *ϕ*_*i*,*j*_^2^ represents the noise variance in the NSST transform decomposition subband. The noise variance can be expressed as follows:

(7) $$\begin{array}{c} \phi_{i,j}^{2}=\frac{\sqrt{\sum_{x=1}^{Z_{l}}\sum_{y=1}^{Z_{l}}J_{i,j}^{\text{NSSST}}\left(x,y\right)J_{i,j}^{\text{NSSST}\#}\left(x,y\right)}}{Z_{j}}, \end{array}$$

where *J*_*i*,*j*_^NSSST^(*x*, *y*) represents the NSST transform coefficient of the *j*-th scale in the *i*-th direction, *J*_*i*,*j*_^NSSST#^(*x*, *y*) is the resurrection yoke of *J*_*i*,*j*_^NSSST^(*x*, *y*), and *Z*_*j*_ represents the length of the subband.

Finally, the threshold of the high-resolution NSST coefficients is solved to obtain the denoising coefficients at various high resolutions. The NSST coefficients after threshold denoising can be expressed as follows:

(8) $$\begin{array}{c} {\overset{⟶}{J}}_{i,j}^{\text{NSSST}}\left(x,y\right)=\left\{\begin{array}{c} J_{i,j}^{\text{NSSST}}\left(x,y\right),\left|J_{i,j}^{\text{NSSST}}\left(x,y\right)\right|\geq S_{i,j}\\ 0 \end{array}\right\}. \end{array}$$

The above is the optimization process of the NSST. A larger threshold value is used at high resolution, and a smaller threshold value is used at lower resolution to effectively filter out the noise at each high resolution.

However, the low-resolution coefficients after the optimization still retain less low-frequency noise, so further processing is necessary. Therefore, the NSST coefficients are combined with the nuclear anisotropic diffusion model to perform anisotropic diffusion denoising on the NSST coefficients of the low-frequency subbands so that the low-frequency noise is filtered out and the low-frequency details are also well preserved. Next, the NSST coefficients substitute the two-dimensional image, and the new nuclear anisotropic diffusion model can be expressed as follows:

(9) $$\begin{array}{c} J^{\text{NSST}}\left(e=0\right)=J^{\text{NSST}}{}_{0},\\ \frac{\partial J^{\text{NSST}}\left(x,y\right)}{\partial e}=\text{Div}\left[c\left(\left\|\nabla \Phi \left(J^{\text{NSST}}\right)\right\|\right)\nabla J^{\text{NSST}}\right],\\ {\left\|\nabla \Phi \left(J^{\text{NSST}}\right)\right\|}_{u}={\left[\frac{\sum_{v\in \lambda_{u}}{\left\|J_{u}^{\text{NSST}}-J_{v}^{\text{NSST}}\right\|}^{2}}{\left|\lambda_{u}\right|}\right]}^{0.5}, \end{array}$$

where *J*^NSST^ represents the NSST coefficient matrix in the low-frequency subband after the ultrasound image is decomposed by NSST, Φ() is the mapping function, ‖∇Φ(*J*^*NSST*^)‖ represents the nuclear gradient modulus in the eigenspace determined by the mapping function, *λ*_*u*_ represents the field of *u*, and |*λ*_*u*_| represents the size of the field. Then, kernel replacement is performed, and the square of the gray difference in a certain characteristic direction in the feature space can be expressed as follows:

(10) $$\begin{array}{c} {\left\|\Phi \left(J_{u}^{\text{NSST}}\right)-\Phi \left(J_{v}\right)\right\|}^{2}=F\left(J_{u}^{\text{NSST}},J_{u}^{\text{NSST}}\right)+F\left(J_{v}^{\text{NSST}},J_{v}^{\text{NSST}}\right)+F\left(J_{u}^{\text{NSST}},J_{v}^{\text{NSST}}\right),\\ {\left\|\nabla \Phi \left(J^{\text{NSST}}\right)\right\|}_{u}={\left[\frac{\sum_{v\in \lambda_{u}}F\left(J_{u}^{\text{NSST}},J_{u}^{\text{NSST}}\right)+F\left(J_{v}^{\text{NSST}},J_{v}^{\text{NSST}}\right)+F\left(J_{u}^{\text{NSST}},J_{u}^{\text{NSST}}\right)}{\left|\lambda_{u}\right|}\right]}^{0.5}. \end{array}$$

To better control the degree of local diffusion, the grayscale and nuclear gradient models are jointly used to control the degree of diffusion of the image. Then, the optimized diffusion equation is as follows:

(11) $$\begin{array}{c} c\left(\left\|\nabla \Phi \left(J^{\text{NSST}}\right)\right\|\right)=\exp\left(-{\left(\frac{\phi_{F}\left\|\nabla \Phi \left(J^{\text{NSST}}\right)\right\|}{4\tau }\right)}^{2}\right), \end{array}$$

where *ϕ*_*F*_^2^ represents the local grayscale variance of the image and *τ* represents the diffusion threshold, expressed as follows:

(12) $$\begin{array}{c} \tau =\text{median}\left(\left\|\nabla \Phi \left(J^{\text{NSST}}\right)\right\|\right)-\text{median}\left(\left\|\nabla \Phi \left(J^{\text{NSST}}\right)\right\|\right), \end{array}$$

where median() represents the median function.

Combining the NSST coefficients with the nuclear anisotropic diffusion model can realize high-quality denoising of ultrasound images.  Figure 3 shows the specific process.

### 2.4. Observation Indicators

Basic information of groups 1 and 2 was recorded, such as the admission age, bilateral stone rate, feeding time, amount of milk taken, and feeding methods (mixed feeding and artificial feeding). Then, groups 1 and 2 were compared for the effective rate (disappearance of stones, reduction of stones, and no change in stones) and prognosis (discharge rate with stones, stone disappearance rate after 1 year, discharge rate with water accumulation, and water disappearance rate after 1 year). Next, the renal function indexes (blood urea nitrogen (BUN) and blood creatinine (Cr)) and serum inflammatory factors (TNF-*α* and C-reactive protein (CRP)) of group 1, group 2, and the healthy control group were recorded after treatment.

### 2.5. Statistical Methods

The data was processed by SPSS19.0 version statistical software, the measurement data were expressed by the mean ± standard deviation (‾*x* ± *s*), and the count data were expressed by the percentage (%). One-way analysis of variance was used for pairwise comparison. The difference was statistically significant at *P* < 0.05.

## 3. Results

### 3.1. Denoising Results

The Lena images and Barbara images with different degrees of Gaussian white noise pollution (noise standard deviations were 5, 15, and 25, resp.) were used as samples, and the original images were all grayscale images with a size of 521 × 521. The anisotropic diffusion denoising algorithm based on LPND, the denoising algorithm based on the traditional NSST transform, and the denoising algorithm based on KDA were introduced to compare with the algorithm of the study. The four algorithms were then compared for the PSNR, SSIM, and EPI [20].

As shown in Figure 4, for the Lena images with different degrees of Gaussian white noise pollution, the PNSR, SSIM, and EPI indicators of the four algorithms all decreased as the noise standard deviation increased. The indexes of PNSR, SSIM, and EPI of the algorithm in this study were always greater than those of LPND, NSST, and KDA, and the difference was statistically significant (*P* < 0.05).

As shown in Figure 5, for the Barbara images with different degrees of Gaussian white noise pollution, the PNSR, SSIM, and EPI of the four algorithms all decreased as the noise standard deviation increased. The PNSR, SSIM, and EPI of the algorithm in this study were always greater than those of the LPND, NSST, and KDA algorithms, and the difference was statistically significant (*P* < 0.05).

### 3.2. The Denoising Effect of the Algorithm for the Ultrasound Images of Children

Figure 6 shows the denoising performance of four algorithms for ultrasound images of renal failure. It was noted that the image noise and artifacts were significantly reduced versus the original image after being processed by the four algorithms, and the image quality was improved. Of the four algorithms, the algorithm in this study demonstrated the best denoising effects, with higher definition and less noise and artifacts.

Further quantitative comparison found (Figure 7) that the PNSR, SSIM, and EPI of the algorithm in this study were significantly greater than those of the LPND, NSST, and KDA algorithms, and the difference was statistically significant (*P* < 0.05).

### 3.3. Comparison of Clinical Data between Group 1 and Group 2

Figure 8 shows the clinical data of the children in groups 1 and 2. It was noted that the admission age of the children in group 1 was significantly younger than that of group 2, the bilateral stone rate was significantly higher than that in group 2, and the difference was statistically significant (*P* < 0.05). There were no statistically significant differences in the feeding time, the amount of milk taken, and the feeding methods of the children in groups 1 and 2 (*P* > 0.05).

Figure 9(a) is an ultrasound image of a child with melamine urinary calculi, and it shows dilated ureter and hyperechoic echo with acoustic shadow, central echo separation, and anechoic area around the kidney.  Figure 9(b) is an image of a child with melamine urinary calculi and renal failure. It was noted that the kidney was slightly enlarged, the cortex was thickened, the cortex and medulla were clearly demarcated, and the medulla contour was obviously enlarged.

### 3.4. Total Effective Rate of Treatment for Children in Groups 1 and 2

It was noted from Figure 10 that, of the 52 children in group 1, the stone disappeared in 25 cases after treatment, the stone was reduced in 20 cases, and the stone remained unchanged in 7 cases. The total effective rate of treatment was 88.46%. Of the 38 cases in group 2, the stone disappeared in 22 cases after treatment, the stone was reduced in 12 cases, and the stone remained unchanged in 4 cases. The total effective rate of treatment was 89.47%. There was no statistically significant difference in the total treatment effective rate between the two groups of children (*P* > 0.05).

### 3.5. Comparison of Prognosis of Children in Groups 1 and 2

Figure 11 shows the prognosis of children in groups 1 and 2. No difference was noted in the rate of discharge with stones, the rate of stone disappearance after 1 year, the rate of discharge with water accumulation, and the water loss rate after 1 year (*P* > 0.05).

### 3.6. Comparison of Renal Function of Children in Group 1, Group 2, and the Healthy Control Group

Figure 12 shows the renal function of children in group 1, group 2, and the healthy control group after treatment. No difference was noted in the blood BUN and blood Cr of the children in group 1, group 2, and the healthy control group after treatment (*P* > 0.05).

### 3.7. Comparison of Serum Inflammatory Factors in Children of Groups 1 and 2 after Treatment with the Healthy Control Group

Figure 13 shows the serum inflammatory factors in children of groups 1 and 2 and the healthy control group after treatment. No difference was noted in the TNF-*α* and CRP levels of children between group 1, group 2, and the healthy control group after treatment (*P* > 0.05).

## 4. Discussion

Acute renal failure is a common kidney disease, and it is associated with many factors, such as changes in human hemodynamics and injury from toxic substances [21]. The clinical manifestations of urinary calculi in children are often atypical and easily confused with other abdominal diseases. If diagnosis and treatment are delayed, it may be complicated by acute kidney failure [22]. In this study, 90 children with melamine urinary calculi were selected as research subjects. Of them, 52 cases were in group 1 (nonrenal failure), and 38 cases were in group 2 (combined with renal failure). In addition, 35 hospitalized children with no history of melamine-contaminated milk feeding during the same period were used as a healthy control. They all underwent ultrasound imaging examination based on the speckle noise algorithm, and the prognosis was analyzed. Firstly, the Lena images and Barbara images with different degrees of Gaussian white noise pollution (noise standard deviations were 5, 15, and 25, resp.) were used as samples. It was found that the PNSR, SSIM, and EPI indicators of the four algorithms all decreased as the noise standard deviation increased. The indexes of PNSR, SSIM, and EPI of the algorithm in this study were always greater than those of LPND, NSST, and KDA, and the difference was statistically significant (*P* < 0.05). This was in line with the research results of Li et al. (2016) [23] that compared with the traditional ultrasonic denoising technology, this algorithm can overcome the contradiction between noise filtering and entry edge reservation, indicating that the algorithm in this study had a good denoising effect on images with different degrees of noise pollution. After the algorithms were applied to ultrasound images of renal failure, it was noted that the image noise and artifacts were significantly reduced versus the original image after being processed by the four algorithms, and the image quality was improved. Of the four algorithms, the algorithm in this study demonstrated the best denoising effects, with higher definition and less noise and artifacts [24].

The clinical data of the children in groups 1 and 2 were compared, and it was found that the admission age of the children in group 1 group was significantly younger than that in group 2, the bilateral stone rate was significantly higher than group 2, and the difference was statistically significant (*P* < 0.05), which indicated that renal failure might be related to the age [25]. Of the 52 children in group 1, the stone disappeared in 25 cases after treatment, the stone was reduced in 20 cases, and the stone remained unchanged in 7 cases. The total effective rate of treatment was 88.46%. Of the 38 cases in group 2, the stone disappeared in 22 cases after treatment, the stone was reduced in 12 cases, and the stone remained unchanged in 4 cases. The total effective rate of treatment was 89.47%. There was no statistically significant difference in the total treatment effective rate between the two groups of children. In this study, hemodialysis was used for children with renal failure, and there was no bleeding or infection during the treatment, and the treatment effect was good. As for the prognosis, no difference was noted in the rate of discharge with stones, the rate of stone disappearance after 1 year, the rate of discharge with water accumulation, and the water loss rate after 1 year (*P* > 0.05). It suggested that children with renal failure had a good prognosis after treatment, and most of the symptoms disappeared or were alleviated [26]. No difference was noted in the blood BUN and blood Cr of the children in group 1, group 2, and the healthy control group after treatment (*P* > 0.05). It suggested that the renal function of children with renal failure recovered after treatment to normal. In terms of the comparison of serum inflammatory factors, no difference was noted in the TNF-*α* and CRP levels of children between group 1, group 2, and the healthy control group after treatment (*P* > 0.05). It also showed that the serum inflammatory factor levels returned to normal after treatment, and the inflammatory response was weakened [27].

## 5. Conclusion

In this study, 90 children with melamine urinary calculi were selected as research subjects. Of them, 52 cases were in group 1 (nonrenal failure), and 38 cases were in group 2 (combined with renal failure). In addition, 35 hospitalized children with no history of melamine-contaminated milk feeding during the same period were used as a healthy control. They all underwent ultrasound imaging examination based on the speckle noise algorithm, and the prognosis was analyzed. The results showed that the denoising algorithm based on ST and KDA model in this study had good denoising effect on ultrasound images than traditional algorithms, with higher definition and less noise and artifacts. It has been proved that the clinical treatment of children with urinary calculi and renal failure is highly effective, the renal function and serum inflammatory factor levels return to the normal range, and the inflammatory response is weakened. However, some limitations in the study should be noted. The sample size is small, which will reduce the power of the study. In the follow-up, an expanded sample size is necessary to strengthen the findings of the study. In conclusion, this study provides good theoretical support for the clinical diagnosis and treatment of urinary calculi complicated with renal failure.

## Figures and Tables

**Figure 1:** Shear wave support frequency domain in the *ℜ*^2^ plane.

**Figure 2:** High- and low-frequency subband processing flow based on NSST transform.

**Figure 3:** Image denoising process based on NSST coefficients and nuclear anisotropic diffusion model.

**Figure 4:** The denoising performance of the four algorithms for Lena images with different degrees of Gaussian white noise pollution: (a) PSNR; (b) SSIM; (c) EPI.^*∗*^The difference compared with the algorithm in this study is statistically significant (*P* < 0.05).

**Figure 5:** The denoising performance of the four algorithms Barbara images with different degrees of Gaussian white noise pollution: (a) PSNR; (b) SSIM; (c) EPI. ^*∗*^The difference compared with the algorithm in this study is statistically significant (*P* < 0.05).

**Figure 6:** Denoising performance of four algorithms on ultrasound images of renal failure. (a)–(e) are the original image, image processed by the LPND algorithm, image processed by the NSST algorithm, image processed by the KDA algorithm, and image processed by the algorithm in this study.

**Figure 7:** The denoising performance of four algorithms on ultrasound images of renal failure. ^*∗*^The difference compared with the algorithm in this study is statistically significant (*P* < 0.05).

**Figure 8:** Comparison of clinical data between groups 1 and 2: (a) the age of admission and the rate of bilateral stones; (b) the feeding time and the amount of milk taken; (c) the feeding methods (mixed feeding and artificial feeding).

**Figure 9:** Ultrasound images of the patients: (a) an ultrasound of a child with melamine urinary calculi; (b) an ultrasound of a child with melamine urinary calculi and renal failure.

**Figure 10:** The total effective rate of treatment for children in groups 1 and 2. The inner circle represented group 1, and the outer circle represented group 2.

**Figure 11:** Comparison of prognosis of children in groups 1 and 2: (a) rate of discharge with stones and rate of stone disappearance after 1 year; (b) rate of discharge with water accumulation and rate of water loss after 1 year.

**Figure 12:** Comparison of kidney function of children in group 1, group 2, and the healthy control group.

**Figure 13:** Comparison of serum inflammatory factors in children of group 1, group 2, and the healthy control group after treatment.

## Data Availability

The data used to support the findings of this study are available from the corresponding author upon request.
